# Vitamin B_2_ Prevents Glucocorticoid-Caused Damage of Blood Vessels in Osteonecrosis of the Femoral Head

**DOI:** 10.1155/2022/4006184

**Published:** 2022-07-06

**Authors:** MinKang Guo, Jian Zhang

**Affiliations:** ^1^Orthopedic Laboratory of Chongqing Medical University, China; ^2^Department of Orthopedics, The First Affiliated Hospital of Chongqing Medical University, China

## Abstract

Osteonecrosis of the femoral head (ONFH) is a disorder that can cause collapse of the femoral head. The damage and dysfunction of femoral head microvascular endothelial cells are related to the pathogenesis of glucocorticoid-induced ONFH. Reports suggest that vitamin B_2_ can promote osteoblast differentiation and prevent low bone mineral density and prevent reperfusion oxidative injury. To explore the effect and possible molecular mechanism of vitamin B_2_ on the ONFH and Human Umbilical Vein Endothelial Cells (HUVECs), we performed a rat model of ONFH by dexamethasone. The rats were randomly divided into four groups: control group, vitamin B_2_ group, dexamethasone group, and dexamethasone combined with vitamin B_2_ treatment group. HUVECs were used to further prove the role and mechanism of vitamin B_2_ in vitro. In patients, according to immunohistochemical and qRT-PCR of the femoral head, the angiogenic capacity of the ONFH femoral head is compromised. In vivo, it showed that vitamin B_2_ could inhibit glucocorticoid-induced ONFH-like changes in rats by suppressing cell apoptosis, promoting the regeneration of blood vessels, and increasing bone mass. According to in vitro results, vitamin B_2_ could induce the migration of HUVECs, enhance the expression of angiogenesis-related factors, and inhibit glucocorticoid-induced apoptosis. The underlying mechanism may be that vitamin B_2_ activates the PI3K signaling pathway. Vitamin B_2_ alleviated dexamethasone-induced ONFH, and vitamin B_2_ could promote the proliferation and migration of HUVECs and inhibit their apoptosis by activating the PI3K/Akt signaling pathway. Vitamin B_2_ may be a potentially effective treatment for ONFH.

## 1. Introduction

Osteonecrosis of the femoral head (ONFH) is a common cause of hip disability among the middle-aged, with bilateral necrosis in 30 to 70 percent of cases, which severely affects patients' life and places a burden on public health finance [1, 2]. Clinically, glucocorticoid (GC) administration is considered the most common cause of ONFH, as 9 to 40 percent of patients treated with glucocorticoids experience ONFH [3, 4]. Specifically, a reduced number of blood vessels and reduced blood supply are considered important mechanisms of ONFH [5]. Presently, nonsurgical treatments for this disease include load protection, drug treatment, and physical therapy [6]. However, the effects of these conservative treatments are uncertain. Currently, surgery is still the main treatment option.

GC induced thrombosis, endothelial cell dysfunction and damage, and endothelial cell apoptosis, which leads to the development of ONFH [7]. Previous research has established that angiogenesis and osteogenesis are closely related [8]. Moreover, GC inhibits the activity of osteoblasts and osteocytes and decreases the number of blood vessels in bones, together leading to bone loss [9]. GC inhibited angiogenesis in bone and inhibited HIF-1*α* transcription and VEGF production in osteoblasts and osteocytes. GC inhibits the expression of VEGF, which is one of the key growth factors regulating vascular development and angiogenesis. VEGF directly regulates the differentiation and function of osteoblasts and osteoclasts [10, 11]. VEGF also exerts direct effects on osteoblasts via BMP produced by endothelial cells [12]. Therefore, drugs that can promote blood vessel formation would be promising for the treatment of ONFH.

Vitamin B_2_ in form of flavin adenine dinucleotide (FAD) and flavin mononucleotide (FMN) participates in redox reactions in the metabolic pathways that are involved in energy production [13, 14]. Perumal et al. demonstrated that lipid peroxidation and reperfusion oxidative injury of mitochondria were possibly prevented by vitamin B_2_ [15]. In a model of hepatocyte ischemia/reperfusion injury, vitamin B_2_ attenuates tissue oxidative/nitrosative stress and inflammatory infiltration and exerts antioxidants and effects after hepatic ischemia/reperfusion, reducing the damage of hepatocytes [16]. Moreover, vitamin B_2_ showed a protective effect in lipopolysaccharide-induced lung injury in rats [17]. Cheung et al. showed that vitamin B_2_ promotes the synthesis of normal extracellular matrix and reduces reactive oxygen species levels in keratoconus [18]. Vitamin B_2_ has an additive effect on osteoblast differentiation induced by ascorbic acid and *β*-glycerophosphate, in which the expression of osteoblast transcription factors (Runx2 and *β*-catenin) is upregulated [19]. Several lines of evidence suggest that adequate intake of vitamin B_2_ can promote osteoblast differentiation and prevent low BMD [20, 21]. Interruption of blood supply is a direct cause of ONFH disease, and vascular endothelial cell injury seriously affects the course of ONFH. It would be interesting if we could protect the vascular endothelial cells by medication and save the ONFH patient from surgery. Thus, we hypothesize that vitamin B_2_ can protect the head of femur from GC damage.

Due to the interconnection of angiogenesis and osteogenesis, as well as the physiological function of vitamin B_2_, we investigated whether vitamin B_2_ can rescue the fate of ONFH in GC-treated rats in vivo. At the same time, we also researched whether vitamin B_2_ inhibits apoptosis and increases angiogenesis with or without GC treatment HUVECs.

## 2. Materials and Methods

### 2.1. Processing of Human Samples

The study was approved by the Research Ethics Committee of the First Affiliated Hospital of Chongqing Medical University. Written informed consent was obtained from each donor and approved by the Institutional Review of the First Affiliated Hospital of Chongqing Medical University.

Our study included 5 ONFH patients and 5 femoral neck fracture (FNF) patients. The inclusion criteria of ONFH patients were as follows: (1) X-ray, magnetic resonance imaging (MRI), and pathological findings consistent with a diagnosis of ONFH; (2) levels 3 or 4 disease according to the association research circulation osseous (ARCO); and (3) patients on high doses (>3 g cumulative) of glucocorticoids. The inclusion criteria of FNF patients were X-ray, MRI, and histologic section diagnosis of femoral neck fracture and no history of medication or surgical treatment within one year. The exclusion criteria for both groups were as follows: patients with a severe endogenous disease such as Paget's disease, metabolic bone disease, metastatic bone cancer, or hyperparathyroidism. And all patients are in the same age group.

### 2.2. Cell Culture

Human umbilical vein endothelial cells (HUVECs) were purchased from the Cell Bank of the Chinese Academy of Sciences. HUVECs were cultured in Roswell Park Memorial Institute (RPMI) 1640 supplemented with 10% fetal bovine serum (Gibco, Grand Island, USA), penicillin (100 U/ml), and streptomycin (100 *μ*g/ml) at 37°C in 5% CO_2_. Dexamethasone was administered at a concentration of 100 *μ*M for the apoptosis experiment and 20 *μ*M for the other cell experiments. The concentration of vitamin B_2_ administered to the cells was 20 *μ*M.

### 2.3. In Vivo Studies

The animal experiments were performed in accordance with a previous study [22]. In brief, forty healthy 8-week-old female Sprague-Dawley (S-D) rats weighing 140 to 160 g were randomly divided into a control group, vitamin B_2_ group (VB_2_), dexamethasone group (DEX), and dexamethasone combined with vitamin B_2_ treatment group (DEX+VB_2_), with 10 rats in each group. The rats in the control group were intramuscularly injected with PBS. The rats in the vitamin B_2_ group were intramuscularly injected with vitamin B_2_ (3 mg/kg/day) on the first three days of each week for 4 weeks. The rats in the dexamethasone group were intramuscularly injected with dexamethasone (20 mg/kg/d) for the first three days of each week for the same time duration. In the DEX+VB_2_ group, the rats were intramuscularly injected with dexamethasone and vitamin B_2_ for the first three days of each week for the same duration. Two months after treatment, the rats were sacrificed, and the femoral heads were isolated for microcomputed tomography (micro-CT) examination and immunohistochemical staining. The investigators who performed micro-CT and immunohistochemistry were unaware of group assignments during the experiment and data analysis.

Micro-CT (Skyscan1174, Bruker, Belgium) scans of the rat femoral heads were obtained. At the end of the scanning, N-Recon software was used for three-dimensional reconstruction of the femoral head, and CT-AN software was used to analyze the osteogenic parameters BV/TV, Tb. N, Tb. Th, and Tb. Sp (BV/TV: bone volume per tissue volume; Tb. N: trabecular number; Tb. Th: trabecular thickness; Tb. Sp, trabecular separation).

### 2.4. Immunohistochemistry (IHC) and TUNEL Staining

Femoral head samples were obtained from patients at the Department of Orthopedics, the First Affiliated Hospital of Chongqing Medical University, and rats. We assessed angiogenic differentiation in necrotic areas of bone tissue of ONFH, and the control specimens were obtained from the same areas. In the IHC staining assay [23], paraffin sections were defatted with xylene, boiled in citrate buffer (pH 6.0) for 15 min, incubated with 3% H_2_O_2_ for 25 min at room temperature in the dark to block endogenous peroxidase, and blocked with normal goat serum. Then, the sections were then incubated with primary antibodies overnight at 4°C in a humidified chamber. After being washed, tissues were covered with secondary antibody (HRP labeled) and incubated for 50 min at room temperature. TUNEL staining was performed as previously described [24], the TDT enzyme, dUTP, and buffer in the TUNEL kit according mix at 1 : 5 : 50 ratio at 37°C for 60 min. Reagent streptavidin-HRP is added to cover the tissue and incubated at 37°C for 30minutes. Cell nuclei were stained with DAPI. Stained tissue was visualized under a Nikon E100 microscope (Nikon DS-U3, Japan).

### 2.5. CCK-8 Assay

Cell Counting Kit-8 (CCK-8, MCE, USA) was used to estimate cell proliferation. As previously reported [25], HUVECs were plated in 96-well plates at a density of 5 × 10^3^ cells/well and processed in groups, with three duplicate wells in each group. When the growth and fusion degree reached 70-80 percent, the cells were treated according to these groups and incubated for 24, 48, or 72 h. The corresponding reagents were added according to the instructions of CCK-8 detection kit, and the absorbance (D) value of each well at 450 nm was detected on a microplate reader.

### 2.6. RNA Isolation and Quantitative PCR (qPCR)

Total RNA was purified from human femoral head tissue, rat femoral head tissue, and HUVECs using TRIzol (Invitrogen, USA) according to the manufacturer's instructions [26]. cDNA was generated from the total RNA extracted from tissues or cells with a reverse transcription reaction kit (TAKARA, Japan). The cDNA was used as a template for subsequent qPCR assays. The forward and reverse primers used in this study are shown in Table 1.

### 2.7. Wound Healing Assay

A wound healing assay was performed as described previously [27]. The cells were plated in 6-well plates. When the cells reached 100% confluence, a scratch was made through the cell layer. The nonadherent cells were removed with PBS. The remaining adherent cells were incubated with serum-free medium in the presence or absence of vitamin B_2_ and dexamethasone to allow cell growth and wound healing. Every 12 h, the cells were photographed with a phase contrast microscope (Olympus, Tokyo, Japan).

### 2.8. Cell Apoptosis Assay

Cell apoptosis was analyzed by flow cytometry [28]. The cells were incubated in serum-free medium in the presence or absence of vitamin B_2_ and dexamethasone for 72 h. The cells were digested with 0.05% EDTA-free trypsin, collected, and washed with PBS twice. The cells were stained with staining Annexin V-FITC (BD Pharmingen, USA) and propidium iodide (BD Pharmingen, USA). The cells were incubated at room temperature for 20 min, and the cell apoptosis rate was assessed on flow cytometer.

### 2.9. Western Blot Assay

Protein expression levels were measured by Western blotting [29]. Briefly, protein was extracted with RIPA lysis buffer (Beyotime, China), and the total protein concentration was determined with a Bicinchoninic Acid (BCA) Protein Assay Kit (Beyotime, China). After electrophoresis, the proteins were transferred to a polyvinylidene difluoride (PVDF) membrane (Millipore Corporation, USA), which was blocked in 5% fat-free milk powder (Boster Biological Technology, China) for 60 min at room temperature. The PVDF membrane was incubated with primary antibody overnight at 4°C. Next, the membrane was washed in TBST and incubated with secondary antibodies for 60 min. Primary antibodies against PI3K (1 : 1000, Abcam), p-PI3K (1 : 1000, Abcam), AKT (1 : 1000, Abcam), p-AKT (1 : 1000, Abcam), VEGF (1 : 1000, Wanleibio), VWF (1 : 1000, Wanleibio), CD31 (1 : 1000, Wanleibio), and GAPDH (Abcam, 1; 2000) were used.

### 2.10. Statistical Analysis

All experiments were performed in triplicate, and the experimental data are presented as mean ± standard deviation (SD). We applied one-way analysis of variance (ANOVA) and Student's *t*-test to analyze the data for each group. Differences were considered statistically significant when *P* values < 0.05.

## 3. Results

### 3.1. Diminished Angiogenesis Capacity in the Femoral Head of ONFH Patients

The general shapes of femoral heads are shown in Figure 1(a), the image on the left shows the femoral head of a femoral neck fracture (FNF) patient, and the image on the right shows the femoral head of a patient with ONFH. In Figure 1(b), the X-ray image shows a change in femoral head density and narrowing of the joint space. In Figure 1(c), the MRI image shows a subchondral fracture with low signal strength. Angiogenesis plays an important role in bone development and regeneration. Thus, we assessed angiogenic differentiation in necrotic areas of bone tissue of ONFH patients, and fracture specimens were obtained from the corresponding areas. Immunohistochemical images showed that the expression of VEGF, critical markers of angiogenesis, was notably decreased in ONFH bone tissue (Figure 1(d)). Meanwhile, the qPCR results showed that the mRNA levels of VEGF, CD31, VWF, ANGPT1, and EMCN were significantly decreased in ONFH bone tissue compared with FNF bone tissue (Figure 1(e)). In summary, these data suggested that vasculogenic capacity was impaired in the femoral heads of ONFH patients.

### 3.2. Vitamin B_2_ Facilitates Bone Formation of Femoral Head In Vivo

To assess the effect of vitamin B_2_ on bone mass and angiogenesis in vivo, the rats were treated according to the corresponding protocol for 8 weeks to establish an ONFH model [22]. Three-dimensional micro-CT images showed that the rat model of ONFH was successfully established. Analysis of the femoral head showed that 60% of the rats injected with dexamethasone developed trabecular changes, including decreased bone volume, trabecular number, and trabecular thickness, an increase in trabecular separation (Figure 2(a)). However, the trend of the dexamethasone-induced decrease in bone mass was rescued by vitamin B_2_ (Figure 2(b)). The immunohistochemical images showed that the expression of OCN significantly declined in the DEX group, showing that dexamethasone inhibits bone formation in the femoral head. In the DEX+VB_2_ group, the bone mass was recovered (Figure 2(c)). The qPCR results showed that the expression of ALP, OCN, BSP, and RUNX2 was significantly downregulated in the DEX group, and vitamin B_2_ restored the expression of ALP, OCN, BSP, and RUNX2 to some extent (Figure 2(d)). These data suggested that vitamin B_2_ probably limits the dexamethasone-induced impairment of osteogenesis in vivo.

### 3.3. Vitamin B_2_ Facilitates Angiogenesis of Femoral Head In Vivo

Immunohistochemical staining showed that the expression of VEGF was significantly decreased in the DEX group and that dexamethasone dramatically inhibited the growth of vascular endothelial cells. In the DEX+VB_2_ group, the viability of vascular endothelial cells and the expression of VEGF was recovered (Figure 3(a)). Consistent with this finding, the qPCR results showed that the expression of VEGF, CD31, VWF, EMCN, and ANGPT1 was significantly downregulated in the DEX group and that vitamin B_2_ restored the expression of angiogenesis factors to some extent (Figure 3(b)) TUNEL staining revealed many more apoptotic cells in the DEX group than in the other groups and showed that vitamin B_2_ inhibited dexamethasone-induced apoptosis to some extent (Figure 3(c)). Collectively, these results confirmed that vitamin B_2_ probably restores angiogenesis after it is impaired by dexamethasone in vivo. We also observed the effect of dexamethasone on the apoptosis of cells in femoral head tissue.

### 3.4. Vitamin B_2_ Promotes the Proliferation and Migration and Inhibits Apoptosis of HUVECs

CCK8 results showed that the proliferation ability of HUVECs was enhanced with increasing vitamin B_2_ concentration in a certain concentration range. When vitamin B_2_ treatment concentration was 20 *μ*mol/L, the proliferation ability of HUVECs was strongest (Figure 4(a)). Dexamethasone significantly inhibited the proliferation ability of HUVECs, and the proliferation ability of HUVECs in the DEX+VB_2_ group was partially restored compared with the DEX group (Figure 4(b)). The above results suggested that dexamethasone inhibited the proliferation of HUVECs, and vitamin B_2_ could partially restore the dexamethasone-induced decrease in the proliferation of HUVECs. The wound healing assay showed that after 72 h, few cells in the DEX group migrated and that more cells migrated in the DEX+VB_2_ group than in the DEX group (Figures 4(c) and 4(d)). This result indicated that vitamin B_2_ prevented the inhibitory effect of dexamethasone on HUVEC migration. Next, a fluorescent conjugated Annexin V antibody was used to detect apoptotic cells due to its high affinity for anionic phospholipid phosphatidylserine on the outer surface of apoptotic cells. The results showed that apoptosis of HUVECs was triggered by dexamethasone and that vitamin B_2_ markedly reversed dexamethasone-induced apoptosis (Figures 4(e) and 4(f)).

### 3.5. Mechanisms of Vitamin B_2_ Rescue the Impaired Angiogenic Function in ONFH

To explore potential mechanisms by which vitamin B_2_ rescues the impaired angiogenic function in ONFH, the qPCR and Western blot were performed. This effect of vitamin B_2_ was further confirmed by its ability to reverse the change in the expression of angiogenesis-related genes VEGF, CD31, ANGPT1, and VWF, which was downregulated by dexamethasone alone (Figure 5(a)). Consistent with the above results, Western blot analysis confirmed that vitamin B_2_ could restore the expression of VEGF, CD31, and VWF in dexamethasone-treated HUVECs (Figure 5(b)). The PI3K/AKT pathway is known to play a key role in numerous cellular functions including proliferation, migration, and metabolism [30]. The PI3K/AKT pathway induces VEGF mRNA transcription and VEGF protein expression which stimulates the formation of blood vessels [31]. The results confirmed that dexamethasone inhibited the levels of p-PI3K, p-Akt, and VEGF, and dexamethasone combined with vitamin B_2_ treatment group increased the expression of p-PI3K, p-Akt, and VEGF which resulted in the activation of the PI3K/Akt signaling pathway (Figure 5(c)). The Western blot results revealed that mechanistically, the PI3K/Akt pathway is important for migration, apoptosis, and expression of angiogenesis-related factors in HUVECs and that vitamin B_2_ is vital in activating this pathway.

## 4. Discussion

ONFH is a common refractory disease in orthopedics, which affects millions of people in China [32]. In the United States, its incidence is estimated at 15,000-20,000 new cases per year [33]. Osteonecrosis is characterized by bone cell death due to impaired blood supply to the bones, and osteonecrosis is most common in the femoral head [34]. The microenvironment of ONFH is closely related to cell proliferation, apoptosis, osteogenic differentiation, and angiogenesis [35]. Seguin et al. [36] showed that ONFH is strongly associated with regional endothelial dysfunction. And vascular endothelial cells play an important role in maintaining this microenvironment. Moreover, previous in vivo and in vitro experiments have provided large amounts of evidence that GC inhibits angiogenesis while also decreasing bone formation and increasing bone resorption [5]. In this study, vitamin B_2_ was found to reduce the negative effects of dexamethasone on angiogenesis-related cytokine expression, bone formation, and apoptosis in vivo experiments.

Numerous studies have suggested that vitamin B_2_ prevents oxidative damage by peroxidation and reperfusion and can promote osteoblast differentiation and treat osteoporosis [37]. Vitamin B_2_ is a water-soluble vitamin, and riboflavin transporter assists its entry into cells [38]. Vitamin B_2_ has an additive effect on ascorbic acid, and *β*-glycerophosphate induced osteogenic differentiation of MC3T3-E1 cells, which is characterized by enhanced alkaline phosphatase activity and promotion of osteogenic differentiation [19]. However, these studies have mainly focused on the effect of vitamin B_2_ on osteoporosis, and there are few studies related to ONFH.

At present, research on ONFH mainly focuses on the balance between osteoblast and osteoclast production [39]. However, femoral head tissue contains a variety of cells, such as mesenchymal stem cells, osteoblasts, and vascular endothelial cells. In the skeletal system, the vascular system is critical for bone development and remodeling and is essential for maintaining healthy bone tissue. Dysregulation of bone-vascular interactions underlies different pathologies [40, 41]. Previous studies have suggested that ONFH is related to angiogenesis-osteogenesis coupling [42, 43]. GC-induced ONFH is closely associated with dysfunction of bone microvascular endothelial cells (BMECs), and dysfunction of BMECs ultimately leads to reduced local blood flow to the femoral head and is thought to be the cause of GC-induced ONFH [44]. VEGF receptor 2 antibody can induce ONFH in the rat with a high incidence [45]. Xu et al. [6] demonstrated that enhancing VEGF-mediated angiogenesis and inhibiting apoptosis prevent bone loss in mouse ONFH. VEGF regulates the proliferation, migration, and vascularization of endothelial cells and is a key inducer of angiogenesis [46]. Maes et al. [47] suggested that VEGF binds angiogenesis and osteoblastic differentiation through its effects on endothelial cells and regulation of osteoblasts, both of which express VEGF receptors. In our study, mRNA and protein expression of both VEGF and CD31 vascular-related genes were substantially higher in the DEX+VB_2_ group compared to the DEX group, and VB_2_ alone also enhanced their expression, in vivo and in vitro. Furthermore, using immunohistochemical techniques, we observed more vessels with endothelial marker expression in rats with GC and VB_2_ administration, which further affirmed our hypothesis.

Endothelial cells can direct osteogenic differentiation of stem cells by activating AKT signaling pathway [48]. In our study, it was further demonstrated that dexamethasone can directly damage endothelial cells, inhibit cell migration, and promote apoptosis, which is consistent with the previous studies [44]. In addition, studies have confirmed that activation of the PI3K/Akt/VEGF signaling pathway promotes angiogenesis in renal cell carcinoma [49]. Li et al. [50] reported that microRNA-126 inhibited the function of HUVEC by inhibiting the expression of EGFL7 and downregulating the PI3K/AKT signaling pathway. And Chen et al. [51] demonstrated that tectorigenin increased the phosphorylation of PI3K and Akt in HUVEC and reduced H_2_O_2_-induced oxidative stress injury. It was found that in HUVEC cells, the protein levels of p-PI3K and p-AKT in the dexamethasone combined with vitamin B_2_ treatment group were significantly higher than those in the dexamethasone treatment group. The increase in phosphorylated proteins is not due to changes in total protein expression, but due to activation of kinases, which can increase the percentage of phosphorylated proteins. In vitro, these data revealed that the PI3K/Akt pathway is important for migration, apoptosis, and expression of angiogenesis-related cytokines in HUVECs and that vitamin B_2_ is vital in activating this pathway. Interesting, recent studies have found that ONFH is regulated by osteoclasts and microRNAs, not sure if the effects of vitamin B_2_ might modulate these activities [52, 53]. And more research will be conducted in the future.

## 5. Conclusions

In this study, an important role of vitamin B_2_ was found. In vivo, vitamin B_2_ increased bone mass in the femoral head, avoided femoral head collapse, decreased GC-induced bone loss, apoptosis of cells, and increased expression of angiogenesis-related genes. Although it does not fully restore the effects of GC on bone, vitamin B_2_ can attenuate the negative effects of dexamethasone on vascular endothelial cells, such as promoting the migration ability of endothelial cells, inhibiting apoptosis, and promoting the expression of angiogenesis-related factors. This study reveals the positive effect of vitamin B_2_ on angiogenesis and provides new ideas for clinical treatment of glucocorticoid-induced ONFH.

## Figures and Tables

**Figure 1:** Diminished vasculogenic capacity in the femoral heads of ONFH patients. The general shapes of femoral heads are shown in (d), the left image is the femoral head of a femoral neck fracture (FNF) patient, and the image on the right is the femoral head of an osteonecrosis of the femoral head (ONFH) patient. (b and c) A radiograph and MRI image of a femoral head. (d) IHC staining of VEGF in femoral head tissue. (e) q-PCR analysis of VEGF, CD31, VWF, ANGPT1, and EMCN in the femoral head. The data are shown as mean ± SD for five separate experiments. ^∗^*P* < 0.05.

**Figure 2:** Vitamin B_2_ facilitates bone formation of femoral head *in vivo.* (a) Reconstructed COR, TRA, SAG, MPR, and 3-DR images in the femoral heads of each group were obtained using micro-CT (COR: coronal; TRA: transverse; SAG: sagittal; MPR: multiplanar reconstruction; 3-DR: three-dimensional reconstruction). (b) Quantitative analysis of the BV/TV, Tb. N, Tb. Th, and Tb. Sp of each group (BV/TV: bone volume per tissue volume; Tb. N; trabecular number; Tb. Th: trabecular thickness; Tb. Sp: trabecular separation). (c) Representative images of OCN staining in the femoral heads of each group. (d) q-PCR analysis of ALP, OCN, BSP, and RUNX2 in the femoral head. Each experiment was done in triplicate. The data are shown as mean ± SD for triplicate. ^∗^*P* < 0.05.

**Figure 3:** Vitamin B_2_ facilitates angiogenesis of femoral head in vivo. (a) Representative images of VEGF staining in the femoral heads of each group. (b) q-PCR analysis of VEGF, CD31, VWF, EMCN, and ANGPT1 in the femoral head. (c) Representative images of TUNEL staining in the femoral heads of each group. And quantification results were analyzed by ImageJ software. Each experiment was done in triplicate. ^∗^*P* < 0.05.

**Figure 4:** Vitamin B_2_ promotes the proliferation and migration and inhibits apoptosis of HUVECs. (a) The effect of different concentrations of vitamin B_2_ on HUVECs proliferation. (b) The change of proliferation ability of HUVECs in the presence or absence of vitamin B_2_ and dexamethasone. (c) Images of the wound healing assay at 72 h showing a larger number of migrated cells in the vitamin B_2_ coincubation group than the DEX group. (d) Quantitative analysis of the assay shown in (c). (e) The population of apoptotic cells was measured by Annexin V/PI staining and flow cytometric analysis. (f) Quantitative analysis of the data shown in (e). Each experiment was done in triplicate. ^∗^*P* < 0.05.

**Figure 5:** Mechanisms of vitamin B_2_ rescue the impaired angiogenic function in ONFH. (a) q-PCR analysis of VEGF, CD31, VWF, and ANGPT1 in HUVECs. (b) Western blot analysis of angiogenesis-associated proteins in HUVECs. (c) Statistical analysis was performed to measure the results in (b). (d) Western blot analysis of PI3K, p-PI3K, AKT, and p-AKT. (e) Statistical analysis was performed to measure the results in (d). Each experiment was done in triplicate. ^∗^*P* < 0.05.

**Table 1:** The quantitative real-time polymerase chain reaction primer sequences.

Species	Genes	Forward primer	Reverse primer
Human	VEGF	GCCTTGCCTTGCTGCTCTACC	GGTCTCGATTGGATGGCAGTAGC
Human	CD31	CGTCAAGCCTCAGCACCAGATG	GCACTCCTTCCACCAACACCTG
Human	ANG	CGCTGCCATTCTGACTCACATAGG	CGTACTCTCACGACAGTTGCCATC
Human	EMCN	TTCAGCAACCAGCCGGTCTTATTC	GGATCTGCCTTCCAGCACATTCG
Human	VWF	GCCGACTTCAACAGGAGCAAGG	GCAGCACCGTGACGTGGATG
Human	GAPDH	GGAGCGAGATCCCTCCAAAAT	GGCTGTTGTCATACTTCTCATGG
Rat	ALP	GTGCCCTGGCGACATGATACTG	TGCGGGACATAAGCGAGTTTCTG
Rat	BSP	AAGCGACGAGGAAGAGGAAGAGG	TTGGTGCTGGTGCCGTTGAC
Rat	OCN	GGACCCTCTCTCTGCTCACTCTG	ACCTTACTGCCCTCCTGCTTGG
Rat	RUNX2	TCCGCCACCACTCACTACCAC	GGAACTGATAGGACGCTGACGAAG
Rat	VEGF	CACGACAGAAGGGGAGCAGAAAG	GGCACACAGGACGGCTTGAAG
Rat	CD31	CAGAGCCAGCATTGTGACCAGTC	CAAGGCGGCAATGACCACTCC
Rat	ANG	TTCTTCGCTGCCATTCTGACTCAC	GCAGTTCCCGTCGTGTTCTGG
Rat	EMCN	GGCTGCTTCAAGTGACTGCTCTC	ATGTCTGGTGTTGTAGCCGATGC
Rat	VWF	CTGGTGGAGCCTCTGGTGGTAG	CACAAGCCTCCTCCGCAAACC
Rat	GAPDH	ATGCCATCACTGCCACTCA	CCTGCTTCACCACCTTCTTG

## Data Availability

The data used to support the findings of this study are available from the corresponding author upon request.

## References

[1] Arbab D., Konig D. P. (2016). Atraumatic femoral head necrosis in adults. *Deutsches Arzteblatt International*.

[2] Grayson W. L., Bunnell B. A., Martin E., Frazier T., Hung B. P., Gimble J. M. (2015). Stromal cells and stem cells in clinical bone regeneration. *Nature Reviews. Endocrinology*.

[3] Weinstein S. R. (2011). Glucocorticoid-induced bone disease. *The New England Journal of Medicine*.

[4] Cui L., Zhuang Q., Lin J. (2016). Multicentric epidemiologic study on six thousand three hundred and ninety five cases of femoral head osteonecrosis in China. *International Orthopaedics*.

[5] Kerachian M. A., Seguin C., Harvey E. J. (2009). Glucocorticoids in osteonecrosis of the femoral head: a new understanding of the mechanisms of action. *The Journal of Steroid Biochemistry and Molecular Biology*.

[6] Xu T., Jin H., Lao Y. (2017). Administration of erythropoietin prevents bone loss in osteonecrosis of the femoral head in mice. *Molecular Medicine Reports*.

[7] Zhang Q., Jin L. V., Jin L. (2018). Role of coagulopathy in glucocorticoid-induced osteonecrosis of the femoral head. *The Journal of International Medical Research*.

[8] Rather H. A., Jhala D., Vasita R. (2019). Dual functional approaches for osteogenesis coupled angiogenesis in bone tissue engineering. *Materials Science and Engineering: C*.

[9] Lane N. E. (2019). Glucocorticoid-induced osteoporosis: new insights into the pathophysiology and treatments. *Current Osteoporosis Reports*.

[10] Hu K., Olsen B. R. (2016). The roles of vascular endothelial growth factor in bone repair and regeneration. *Bone*.

[11] Hu K., Olsen B. R. (2017). Vascular endothelial growth factor control mechanisms in skeletal growth and repair. *Developmental Dynamics*.

[12] Hankenson K. D., Gagne K., Shaughnessy M. (2015). Extracellular signaling molecules to promote fracture healing and bone regeneration. *Advanced Drug Delivery Reviews*.

[13] Thakur K., Tomar S. K., Singh A. K., Mandal S., Arora S. (2016). Riboflavin and health: a review of recent human research. *Critical Reviews in Food Science and Nutrition*.

[14] Suwannasom N., Kao I., Pruß A., Georgieva R., Bäumler H. (2020). Riboflavin: the health benefits of a forgotten natural vitamin. *International Journal of Molecular Sciences*.

[15] Perumal S. S., Shanthi P., Sachdanandam P. (2005). Augmented efficacy of tamoxifen in rat breast tumorigenesis when gavaged along with riboflavin, niacin, and CoQ10: effects on lipid peroxidation and antioxidants in mitochondria. *Chemico-Biological Interactions*.

[16] Sanches S. C., Ramalho L., Mendes-Braz M. (2014). Riboflavin (vitamin B-2) reduces hepatocellular injury following liver ischaemia and reperfusion in mice. *Food and Chemical Toxicology*.

[17] Al-Harbi N. O., Imam F., Nadeem A. (2015). Riboflavin attenuates lipopolysaccharide-induced lung injury in rats. *Toxicology Mechanisms and Methods*.

[18] Cheung I., McGhee C., Sherwin T. (2014). Beneficial effect of the antioxidant riboflavin on gene expression of extracellular matrix elements, antioxidants and oxidases in keratoconic stromal cells. *Clinical & Experimental Optometry*.

[19] Neto A. H. C., Yano C. L., Paredes-Gamero E. J. (2010). Riboflavin and photoproducts in MC3T3-E1 differentiation. *Toxicology In Vitro*.

[20] Clarke M., Ward M., Dickey W. (2015). B-vitamin status in relation to bone mineral density in treated celiac disease patients. *Scandinavian Journal of Gastroenterology*.

[21] Yazdanpanah N., Uitterlinden A. G., Zillikens M. C. (2008). Low dietary riboflavin but not folate predicts increased fracture risk in postmenopausal women homozygous for the MTHFR 677 T allele. *Journal of Bone and Mineral Research*.

[22] Zhu W., Guo M., Yang W. (2020). CD41-deficient exosomes from non-traumatic femoral head necrosis tissues impair osteogenic differentiation and migration of mesenchymal stem cells. *Cell Death & Disease*.

[23] Xiao P., Zhu Z., Du C. (2021). Silencing Smad7 potentiates BMP2-induced chondrogenic differentiation and inhibits endochondral ossification in human synovial-derived mesenchymal stromal cells. *Stem Cell Research & Therapy*.

[24] He W., Ying-Fu L., Wang H., Peng Y. P. (2019). Delayed treatment of *α*5 GABAA receptor inverse agonist improves functional recovery by enhancing neurogenesis after cerebral ischemia-reperfusion injury in rat MCAO model. *Scientific Reports*.

[25] Zhu P., Zhou K., Lu S., Bai Y., Qi R., Zhang S. (2020). Modulation of aryl hydrocarbon receptor inhibits esophageal squamous cell carcinoma progression by repressing COX2/PGE2/STAT3 axis. *Journal of Cell Communication and Signaling*.

[26] Sun Y., Kim E. J., Felt S. A. (2019). A specific sequence in the genome of respiratory syncytial virus regulates the generation of copy-back defective viral genomes. *PLoS Pathogens*.

[27] Wang J., Cheng P., Pavlyukov M. S. (2020). Targeting NEK2 attenuates glioblastoma growth and radioresistance by destabilizing histone methyltransferase EZH2. *The Journal of Clinical Investigation*.

[28] Shang A., Gu C., Wang W. (2020). Exosomal circPACRGL promotes progression of colorectal cancer via the miR-142-3p/miR-506-3p- TGF-*β*1 axis. *Molecular Cancer*.

[29] Kondo H., Ratcliffe C., Hooper S. (2021). Single-cell resolved imaging reveals intra-tumor heterogeneity in glycolysis, transitions between metabolic states, and their regulatory mechanisms. *Cell Reports*.

[30] Bader A. G., Kang S., Zhao L., Vogt P. K. (2005). Oncogenic PI3K deregulates transcription and translation. *Nature Reviews Cancer*.

[31] Karar J., Maity A. (2011). I3K/AKT/mTOR pathway in angiogenesis. *Frontiers in Molecular Neuroscience*.

[32] Zhao D., Zhang F., Wang B. (2020). Guidelines for clinical diagnosis and treatment of osteonecrosis of the femoral head in adults (2019 version). *Journal of Orthopaedic Translation*.

[33] Chughtai M., Piuzzi N. S., Khlopas A., Jones L. C., Goodman S. B., Mont M. A. (2017). An evidence-based guide to the treatment of osteonecrosis of the femoral head. *The bone & joint journal*.

[34] Petek D., Hannouche D., Suva D. (2019). Osteonecrosis of the femoral head: pathophysiology and current concepts of treatment. *EFORT Open Reviews*.

[35] Gillet C., Dalla Valle A., Gaspard N. (2017). Osteonecrosis of the femoral head: lipotoxicity exacerbation in MSC and modifications of the bone marrow fluid. *Endocrinology*.

[36] Seguin C., Kassis J., Busque L. (2008). Non-traumatic necrosis of bone (osteonecrosis) is associated with endothelial cell activation but not thrombophilia. *Rheumatology*.

[37] Saedisomeolia A., Ashoori M. (2018). Riboflavin in human health: a review of current evidences. *Advances in Food and Nutrition Research*.

[38] Jaeger B., Bosch A. M. (2016). Clinical presentation and outcome of riboflavin transporter deficiency: mini review after five years of experience. *Journal of Inherited Metabolic Disease*.

[39] Weinstein R. S., Hogan E. A., Borrelli M. J., Liachenko S., O'Brien C. A., Manolagas S. C. (2017). The pathophysiological sequence of glucocorticoid-induced osteonecrosis of the femoral head in male mice. *Endocrinology*.

[40] Marrella A., Lee T. Y., Lee D. H. (2018). Engineering vascularized and innervated bone biomaterials for improved skeletal tissue regeneration. *Materials Today*.

[41] Pirosa A., Gottardi R., Alexander P. G., Tuan R. S. (2018). Engineering in-vitro stem cell-based vascularized bone models for drug screening and predictive toxicology. *Stem Cell Research & Therapy*.

[42] Zhu S., Bennett S., Kuek V. (2020). Endothelial cells produce angiocrine factors to regulate bone and cartilage via versatile mechanisms. *Theranostics*.

[43] Chim S. M., Tickner J., Chow S. T. (2013). Angiogenic factors in bone local environment. *Cytokine & Growth Factor Reviews*.

[44] Yu H., Liu P., Zuo W. (2020). Decreased angiogenic and increased apoptotic activities of bone microvascular endothelial cells in patients with glucocorticoid-induced osteonecrosis of the femoral head. *BMC Musculoskeletal Disorders*.

[45] Gao Y. S., Wang H. F., Ding H., Zhang C. Q. (2013). A novel rat model of osteonecrosis of the femoral head induced by periarticular injection of vascular endothelial growth factor receptor 2 antibody. *Journal of Surgical Research*.

[46] Eshkar-Oren I., Viukov S. V., Salameh S. (2009). The forming limb skeleton serves as a signaling center for limb vasculature patterning via regulation of Vegf. *Development*.

[47] Maes C., Goossens S., Bartunkova S. (2010). Increased skeletal VEGF enhances *β*-catenin activity and results in excessively ossified bones. *The EMBO Journal*.

[48] Tsai T. L., Wang B., Squire M. W., Guo L. W., Li W. J. (2015). Endothelial cells direct human mesenchymal stem cells for osteo- and chondro-lineage differentiation through endothelin-1 and AKT signaling. *Stem Cell Research & Therapy*.

[49] Di J., Gao K., Qu D., Wu Y., Yang J., Zheng J. (2017). Rap2B promotes angiogenesis via PI3K/AKT/VEGF signaling pathway in human renal cell carcinoma. *Tumor Biology*.

[50] Li Q., Cheng K., Wang A. Y. (2019). MicroRNA-126 inhibits tube formation of HUVECs by interacting with EGFL7 and down-regulating PI3K/AKT signaling pathway. *Biomedicine & Pharmacotherapy*.

[51] Chen X., Zhang W., Sun L., Lian Y. (2021). Tectorigenin protect HUVECs from H_2_O_2_-induced oxidative stress injury by regulating PI3K/Akt pathway. *Tissue and Cell*.

[52] Chen K., Liu Y., He J. (2020). Steroid-induced osteonecrosis of the femoral head reveals enhanced reactive oxygen species and hyperactive osteoclasts. *International Journal of Biological Sciences*.

[53] Hong G., Han X., He W. (2019). Analysis of circulating microRNAs aberrantly expressed in alcohol-induced osteonecrosis of femoral head. *Scientific Reports*.

